# The influence of transgenic (*Bt*) and non-transgenic (non-*Bt*) cotton mulches on weed dynamics, soil properties and productivity of different winter crops

This article has been retracted.

**DOI:** 10.1371/journal.pone.0238716

**Published:** 2020-09-04

**Authors:** Muhammad Waseem Riaz Marral, Muhammad Bismillah Khan, Fiaz Ahmad, Shahid Farooq, Mubshar Hussain

**Affiliations:** 1 Department of Agronomy, Bahauddin Zakariya University, Multan, Pakistan; 2 Physiology/Chemistry Section, Central Cotton Research Institute, Multan, Pakistan; 3 Department of Agronomy, Ghazi University, Dera Ghazi Khan, Pakistan; 4 Agriculture Discipline, College of Science, Health, Engineering and Education, Murdoch University, Murdoch, WA, Australia; Omer Halisdemir Universitesi, TURKEY

## Abstract

The introduction of transgenic cotton (*Bt*-cotton) for controlling bollworms has resulted in increased production; however, the residual effects of mulches from *Bt-*cotton are poorly understood. Therefore, the current study evaluated the impact of *Bt* and non-*Bt* cotton mulches on soil properties, weed dynamics and yield of winter crops sown after cotton. Three different winter crops, i.e., wheat (*Triticum aestivum* L.), canola (*Brassica napus* L.) and Egyptian clover (*Trifolium alexandrinum* L.) and two mulch types, i.e., *Bt* mulch (obtained from *Bt*-cotton cultivars, i.e., ‘CIM-616’ and ‘GH-Mubarik’) and non-*Bt* mulch (obtained from non-*Bt* cultivars, i.e., ‘CIM-620’ and ‘N-414’) were included in the study. The mulches were applied at a rate of 2 t ha^-1^ before planting the winter crops. The *Bt* and non-*Bt* mulches differentially affected soil properties, weed dynamics and productivity of winter crops. The non-*Bt* mulches decreased the soil bulk density and penetration resistance, while increased the soil porosity. Wheat crop increased the soil porosity, pH, available N and soil organic matter content. Overall, non-*Bt* mulches improved the productivity of winter crops compared with *Bt* mulches. The toxins released by *Bt* mulches lowered the weed density; however, it negatively influenced soil properties (bulk density and available nitrogen) and productivity of winter crops. Therefore, appropriate crop rotation measures may be opted for the soils cultivated with *Bt*-cotton to conserve soil and achieve yield sustainability for the crops sown after cotton. Nonetheless, non-*Bt* mulches can be used for improving soil properties and productivity of winter crops.

## Introduction

Cotton (*Gossypium hirsutum* L.) is a dual-purpose crop, globally cultivated for its high-quality fiber and oil. It was cultivated on 33.1 million hectares around the world, which produced 136 million bales during 2019 [1]. Cotton is a cash crop in Pakistan and is ranked 2^nd^ after wheat in terms of cultivation area [2]. It is generally sown in the country in different cropping systems, including cotton-wheat (*Triticum aestivum* L.), cotton-chickpea (*Cicer arietinum* L.) cotton-mustard (*Brassica nigra* L.), cotton-Egyptian-clover (*Trifolium alexandrinum* L.) and cotton-lentil (*Lens culinaris* L.) etc. [3]. Numerous insect pests (>1000) attack cotton crop, of which lepidopterans are considered the most dangerous due to their feeding on leaves and bolls [4]. Genetically-modified transgenic insect-resistant cotton (hereafter referred as *Bt*-cotton) was developed to control lepidopteran pests, especially bollworms [5]. The Gram-positive bacterium *Bacillus thuringiensis* produces >200 *Bt* toxins, each of which kills different insects. The *Bt-*cotton has been equipped with the gene coding for *Bt* toxin as a transgene, which enabled it to produce insecticide in the tissues [6]. The sporulation of *Bt* produces large parasporal proteinaceous crystalline inclusions (*Cry* toxins), which kill the insects eating them [6].

Pakistan has undergone remarkable progress in the development of *Bt*-cotton cultivars and numerous new *Bt* cultivars have been developed and approved in the country during the last decade [7–9]. This development has led to the reduction in area under cultivation of conventional (non-*Bt*) cultivars, while *Bt* cultivars have witnessed an increase in the area under cultivation [7, 10]. Genetically modified (GM) crops are cultivated on an area of 181.5 Mha globally and their area under cultivation is increasing by 3–4% each year [11]. Several studies have indicated that continuously growing GM crops on the same soil results in the addition and absorption of *Bt* toxins to the soil [12–17]. These findings indicated that growing *Bt*-cotton cultivars year after year on the same soil will affect the soil properties [16, 17], weed infestation [18, 19] and performance of the crops following cotton [20–22] due to the release and absorption of *Bt* toxins. Nonetheless, growing non-*Bt* cotton cultivars would not exert these impacts due to the absence of *Bt* toxins.

The absorption of *Bt* toxins in the soil activates different soil enzymes, including urease, phosphomonoesterase and invertase, while inhibits arylsulfatase activity [23]. The increased enzyme activities stimulate microbial activity [17]. Moreover, frequent cultivation of *Bt*-cotton cultivars on the same soil significantly influences the soil nutritional status [24]. The cultivation of *Bt*-cotton cultivars decreases nitrogen (N) and potassium (K), while increases zinc (Zn) and phosphorus (P) contents in the soil [25, 26]. This indicates that toxins from *Bt*-cotton cultivars affect chemical composition of root zone and crop residues, which alter ecosystem functioning and plant growth [27]. Moreover, Strandberg et al. [19] revealed that growing transgenic, herbicide tolerant fodder beet cultivars significantly altered weed communities. However, Bai et al. [18] reported no change in the weed community in response to *Bt*-cotton cultivation.

The performance of winter crops sown after cotton [i.e., wheat, barley (*Hordeum vulgare* L.) and mustard] is not affected by herbicide-tolerant *Bt* cultivars [20]. Similarly, crops sown after *Bt*-corn [i.e., carrot (*Daucus carota* subsp. *sativus* (Hoffm.) Schübl. & G. Martens), radish (*Raphanus raphanistrum* subsp. *sativus* (L.) Domin) and turnip (*Brassica rapa* var. *rapa* L.)] were not affected by the toxins released by *Bt*-corn. Nonetheless, *Bt*-corn mulching did not accumulate any toxins [21, 22]. Different *Bt*-cotton cultivars have dissimilar potential to express *Cry1Ac* protein in soils [28, 29] and its concentration declines as the plant growth progresses [22].

Different mulches are used in various crops grown in semi-arid countries like Pakistan to conserve soil moisture, manage weeds and increase soil nutritional status [30–34]. The mulch materials are costly and incur heavy production costs. The use of natural mulches decreases production cost with crop residues’ management advantage. Since the mulches did not affect the performance of crops [21, 22], these can be effectively used for sustainable agriculture. Cotton produces significant amount of biomass, which can be used as mulch in the crops following it. However, a thorough testing of the impacts of cotton mulches on soil properties and productivity of crops is needed.

Several studies have investigated the impacts of residue incorporation of *Bt*-cotton on soil properties [35–37], weed dynamics [18] and crop performance [21, 22]. However, limited studies have tested these impacts collectively. Nonetheless, the *Bt* and non-*Bt* cotton cultivars’ mulches have been rarely tested in this regard. Therefore, the current study was conducted to investigate the impact of *Bt* and non-*Bt* cotton mulches on soil properties, weed dynamics and productivity of winter crops. Hence, the main aim of the study was to quantify the effects of *Bt* and non-*Bt* mulches on soil properties, weed dynamics and productivity of winter crops.

## Materials and methods

### Experimental site and soil

The current study was conducted at Central Cotton Research Institute, Multan (longitude 30.2°N, 71.43°E, and at altitude of 122 meters above sea level), Pakistan during 2016–17 and 2017–2018. The soil of the experimental site was analyzed before sowing and after harvesting of winter crops in order to assess the nutrient dynamics and physiochemical characteristics. The results of the soil analysis before sowing are given in this section (Table 1), while those of after-harvest are presented in the results section. Similarly, weather data collected at the experimental site are given in Table 2.

**Table 1:** Physiochemical characteristics of experimental soil before initiation of the experiment during both the years of study.

Soil determination	Unit	Years			Unit	Years	
		2016–17	2017–18			2016–17	2017–18
Chemical Analysis				Physical analysis			
Organic matter content	%	0.59	0.56	Silt	%	54.15	54.00
Total nitrogen (N)	%	0.06	0.06	Sand	%	25.75	26.10
Available phosphorus (P)	mg kg^-1^	9.01	9.04	Clay	%	20.10	19.90
Available potassium (K)	mg kg^-1^	245.15	249.15	Textural class		Silty-clay	Silty-clay
pH		8.17	8.19				
EC	dS m^-1^	4.96	5.00				

**Table 2:** Weather data of experimental site during both years of the study.

Month	Temperature (ºC)	Relative humidity (%)	Sunshine (hours)	Total rainfall (mm)	Temperature (ºC)	Relative humidity (%)	Sunshine (hours)	Total rainfall (mm)
2016–17					2017–18			
May	34.3	74.3	5.9	2.0	34.0	63.0	4.8	0.1
June	35.4	69.1	3.4	4.0	33.1	74.9	4.5	45.6
July	33.0	73.0	7.0	36.2	33.6	73.0	7.2	4.9
August	31.6	84.6	7.0	109.0	31.8	85.2	7.7	3.0
September	30.5	82.6	8.1	4.0	30.6	77.0	8.0	10.0
October	26.9	68.8	7.0	0.0	27.0	77.5	7.4	0.0
November	19.9	69.6	2.3	0.0	18.0	81.4	3.7	4.2
December	16.4	78.2	3.5	0.0	14.6	74.9	5.2	16.0
January	12.7	79.4	3.3	11.7	13.6	83.0	4.4	0.0
February	16.4	77.0	6.4	11.0	17.5	75.4	4.9	6.8
March	21.7	68.3	6.3	0.0	23.5	70.9	7.2	0.0
April	30.0	53.5	6.3	5.7	29.5	56.7	5.4	3.0

Source: Central Cotton Research Institute, Multan, Pakistan. The values are monthly averages

### Experimental details

Two *Bt*-cotton cultivars (i.e., CIM-616 and GH-Mubarik) and two non-*Bt* cultivars (i.e., CIM-620 and N-414) were used as mulch sources. The seeds of these cultivars were procured from Central Cotton Research Institute, Multan, Pakistan. Three winter crops, i.e., wheat (cultivar ‘Galaxy-2013’), Egyptian-clover (cultivar ‘Anmol berseem’) and canola (*Brassica napus* L., cultivar ‘Hyola-40’) were used in the experiments to assess the impact of *Bt* and non-*Bt* mulches on their productivity, weed dynamics and soil properties. The seeds of wheat, canola and Egyptian-clover were procured from Ayub Agriculture Research Institute, Faisalabad, Pakistan. The mulches were applied at the rate of 2 t ha^-1^ after seedbed preparation and prior to sowing. For mulch preparation, sticks along with dried leaves and bolls were collected after last picking. The sticks were dried and chopped into small pieces (regarded as mulch) for use in the experiment. The experiment was laid out in randomized complete block design (RCBD) with factorial arrangement in plots measuring 5 × 3 m (15 m^2^) with three replications. The mulches were considered as main plots, whereas winter crops were randomized in sub-plots.

### Crop husbandry

A pre-soaking irrigation of ~10 cm was applied to the experimental fields before preparing the seedbed. When soil reached workable moisture level, seedbeds were prepared according to the nature of each crop. All other agronomic and cultural activities were kept uniform to control insect pests and diseases. Details regarding crop husbandry practices for different crops included in the study are given in Table 3.

**Table 3:** Details regarding planting time, seed rate, fertilizer application and harvesting time of winter crops sown in both years of the study.

Crop	Cultivar	Planting time	Seed rate (kg ha^-1^)	Fertilizer NPK (kg ha^-1^)	R × R (cm)	P × P (cm)	Harvesting Time
**Wheat**	Galaxy-2013	11 and 13 November during 1^st^ and 2^nd^ year, respectively	125	130-100-62	25	-	21 and 24 April during 1^st^ and 2^nd^ year, respectively
**Canola**	Hyola-420		5	90-60-50	30	4–5	11 and 12 April during 1^st^ and 2^nd^ year, respectively
**Egyptian clover**	Anmol berseem		20–25	22-115-0	-	-	Last cutting 25 and 26 April during 1^st^ and 2^nd^ year, respectively

R × R = row-to-row distance, P × P = plant-to-plant distance,— = no P × P or R × R distance was maintained as recommended for the respective crop

### Procedures to record observations

#### Soil properties

Soil samples were taken from five different locations within each experimental unit from 0–30 cm depth with the help of a soil auger. These samples were mixed to get a composite sample. The collected samples were dried and passed through a 2 mm sieve for conducting different analyses. Soil bulk density, particle density and total porosity were measured following Blake [38]. Soil penetration resistance (MPa) was determined by a hand-pushing electronic cone penetrometer. Digital EC meter and pH meter were used to measure soil EC (dS m^-1^) and pH, respectively following the standard methods described by Dellavalle [39]. Soil N concentration (N-NO_3_ and N-NH_4_) was measured according to Houba et al. [40]. Total nitrogen was measured spectrophotometrically with a segmented-flow system. The phosphorus was determined by vanadomolybdate method, potassium by flame photometry, and zinc and iron were determined using an atomic absorption spectrophotometer [41]. The organic matter content (%) was measured using loss-on-ignition protocol as introduced by Hoogsteen et al. [42].

#### Weed dynamics in different winter crops

Weed infestation was evaluated 45 days after sowing (DAS) of each winter crop. Total weed density was regarded as weed dynamics. The procedures of LaMastus and Shaw [43] and Onen et al. [44] were followed to record total weed density. Briefly, l m^2^ quadrate was randomly placed at three different locations in each experimental unit and number of weed species present in the quadrate were counted. The weed species in all quadrates of each experimental unit were added to get total weed density.

### Morphological and yield-related parameters of winter crop

#### Wheat

Data on plant height, number of productive tillers, spike length, total numbers of spikelets, number of grains per spike and 1000-grain weight (g) were recorded. The heights of 10 randomly selected plants from each experimental unit were measured with the help of a measuring tape and averaged. The number of spike bearing tillers around the mother tiller of ten randomly selected plants from each experimental unit were counted and averaged to record number of productive tillers. The length of ten randomly selected spikes from each experimental unit was measured and averaged. Similarly, number of spikelets and grains present in twenty randomly selected plants were carefully counted and averaged. Three random sample of 1000 grains were taken form each seed lot of the experimental units, weighed and averaged to record 1000-grain weight. Whole plot was harvested and threshed manually after drying to calculate grain, straw and biological yields. The yields (biological, grain and straw) were converted into t ha^-1^ by unitary method. Harvest index (HI) was taken as ratio of grain yield to biological yield expressed in percentage.

#### Canola

All plants present in quadrate (1×1 m) at maturity were counted to determine plant population. The average height (cm) of ten randomly selected plants was measured at maturity from the soil level to the tip of the plant. Three plants from each replication of each experimental unit were used to count the number of siliques per plant. The siliques were dried and weighed. The pods were manually threshed and number of seeds were counted. The weight (g) of 1000-seed from randomly sampled seeds per plot was measured on an electronic balance. The mature crop was harvested from plots, sundried and threshed manually to separate seed from chaff to record seed yield per plot, which was converted into kg ha^-1^. The HI was calculated as described for the wheat crop.

#### Egyptian-clover

The plants present in 1 m^2^ area from three different places in each replication of each experimental unit were counted to record plant population. The average height of ten randomly selected plants was measured at maturity from the soil level to the tip of the plant. The plants of each cutting from three randomly selected areas of 1 m^2^ in each experimental unit were taken, then oven dried. The dried plants were weighed and converted into kg ha^-1^. At each forage cut, all plants within the plot were harvested, weighed and averaged. The yields of all the cuts were converted to green forage yield (t/ha). Crude protein was measured by near-infrared spectroscopy following Jafari et al. [45].

### Statistical analysis

The collected data were tested for normality by Shapiro-Wilk normality test [46], which indicated that some of the parameters had non-normal distribution. Therefore, non-normally distributed parameters were transformed by Arcsine transformation technique to meet the normality assumption of Analysis of Variance (ANOVA). The difference among experimental years was tested by paired *t* test, which indicated significant differences among years. Therefore, the data of each year were analyzed and presented separately. Two-way ANOVA was used to test the significance in the dataset [47]. Least significant difference test at 5% probability was used as post-hoc test to separate the means where ANOVA indicated significant differences. All analysis were performed on SPSS software version 21 [48]. All the individual and interactive effects were significant for most of the measured variables; therefore, only interactions among mulches and winter crops were presented and interpreted.

## Results

### Soil physical properties

Different mulch types and winter crops significantly affected bulk density, porosity and penetration resistance, whereas had non-significant effect on particle density during both years (Table 4).

**Table 4:** The impact of different mulch types and winter crops on soil bulk and particle densities, soil porosity and soil penetration resistance.

Mulch type	2016–17			2017–18		
	Wheat	Egyptian clover	Canola	Wheat	Egyptian clover	Canola
	**Soil bulk density (g cm**^**-3**^**)**					
CIM-616*	1.460 ab	1.447 cd	1.450 bcd	1.480 a	1.460 cd	1.460 cd
GH-Mubarik*	1.460 ab	1.443 d	1.450 bcd	1.480 a	1.460 cd	1.460 cd
CIM-620**	1.467 a	1.447 cd	1.457 abc	1.467 bc	1.457 cd	1.453 d
N-414**	1.453 bcd	1.450 bcd	1.450 bcd	1.477 ab	1.453 d	1.450 d
**LSD** (**p ≤ 0.05**)	**0.010**			**0.010**		
	**Soil particle density (g cm**^**-3**^**)**					
CIM-616*	2.59	2.50	2.58	2.71	2.61	2.68
GH-Mubarik*	2.66	2.53	2.65	2.75	2.61	2.65
CIM-620**	2.61	2.64	2.60	2.67	2.63	2.65
N-414**	2.63	2.58	2.69	2.66	2.59	2.63
**LSD** (**p ≤ 0.05**)	**NS**			**NS**		
	**Soil porosity (%)**					
CIM-616*	43.81bcd	42.26 d	43.70 bcd	45.66 ab	44.14 bc	45.56 abc
GH-Mubarik*	45.26 ab	43.14 cd	45.29 ab	46.26 a	44.19 bc	44.86 abc
CIM-620**	43.96 bc	45.20 ab	44.12 bc	45.24 abc	44.62 bc	45.29 abc
N-414**	44.96 ab	43.88 bcd	46.22 a	44.59 bc	43.98 c	44.95 abc
**LSD** (**p ≤ 0.05**)	**1.69**			**1.6**		
	**Soil penetration resistance (MPa)**					
CIM-616*	1.733 cd	1.717 f	1.747 a	1.710 bc	1.703 bcd	1.717 ab
GH-Mubarik*	1.747 a	1.727 de	1.747 a	1.713 ab	1.697 cde	1.717 ab
CIM-620**	1.743 ab	1.723 ef	1.737 bc	1.717 ab	1.690 de	1.703 bcd
N-414**	1.737 bc	1.733 cd	1.743 ab	1.727 a	1.683 e	1.703 bcd
**LSD** (**p ≤ 0.05**)	**0.0097**			**0.01**		

* = *Bt* cultivars

** = non-*Bt* cultivars, Means followed by varying letters for an experimental year differ at significantly (p ≤0.05) from each other, NS = Non-significant

Wheat crop with non-*Bt* mulch during 1^st^ year and with *Bt* mulch during 2^nd^ year had the highest bulk density, whereas lowest values were noted for Egyptian-clover with *Bt* mulch and canola with non-*Bt* mulch during 1^st^ and 2^nd^ year, respectively (Table 4). Contrastingly, particle density was not altered by different mulch types and winter crops during both the years. The highest porosity was noted for canola crop with non-*Bt* mulch during 1^st^ year and wheat crop with *Bt* mulch during 2^nd^ year. The lowest porosity was recorded for Egyptian-clover with *Bt* and non-*Bt* mulch during 1^st^ and 2^nd^ year, respectively (Table 4). Wheat and canola crops with *Bt* mulch during 1^st^ year and wheat crop with non-*Bt* mulch during 2^nd^ year had the highest penetration resistance. The lowest penetration resistance was recorded for Egyptian-clover with *Bt* and non-*Bt* mulch during 1^st^ and 2^nd^ year, respectively (Table 4).

### Soil chemical properties

Different mulch types and winter crops significantly altered different soil chemical properties, i.e., EC, pH, available N, available P, available K, available Zn and available iron (Fe) during both years, except non-significant effect on available K during 2^nd^ year (Table 5).

**Table 5:** The impact of different mulch types and winter crops on chemical properties of soil.

Mulch types	2016–17			2017–18		
	Wheat	Egyptian clover	Canola	Wheat	Egyptian clover	Canola
	**Electric conductivity (dS m**^**-1**^**)**					
CIM-616*	5.357 abc	5.407 ab	5.340 bcd	5.307 abc	5.317 ab	5.247 bcd
GH-Mubarik*	5.367 abc	5.433 a	5.400 ab	5.300 abcd	5.357 a	5.323 ab
CIM-620**	5.267 d	5.343 bcd	5.303 cd	5.217 d	5.283 abcd	5.230 cd
N-414**	5.290 cd	5.333 bcd	5.290 cd	5.240 bcd	5.257 bcd	5.227 cd
**LSD** (**p ≤ 0.05**)	**0.087**			**0.084**		
**pH**						
CIM-616*	8.32 a	8.29 ab	8.24 ab	8.25 ab	8.23 abc	8.19 bc
GH-Mubarik*	8.32 a	8.29 ab	8.24 ab	8.26 a	8.24 abc	8.22 abc
CIM-620**	8.24 ab	8.27 ab	8.22 b	8.22 abc	8.22 abc	8.17 c
N-414**	8.27 ab	8.26 ab	8.29 ab	8.23 abc	8.24 ab	8.25 ab
**LSD** (**p ≤ 0.05**)	**0.08**			**0.07**		
**Available nitrogen (mg kg**^**-1**^**)**						
CIM-616*	0.080 ab	0.073 abcd	0.073 abcd	0.087 a	0.080 ab	0.073 bc
GH-Mubarik*	0.070 bcd	0.063 cd	0.063 cd	0.080 ab	0.067 c	0.063 c
CIM-620**	0.087 a	0.077 abc	0.073 abcd	0.087 a	0.080 ab	0.073 bc
N-414**	0.077 abc	0.067 bcd	0.060 d	0.087 a	0.070 bc	0.067 c
**LSD** (**p ≤ 0.05**)	**0.016**			**0.013**		
	**Available phosphorous (mg kg**^**-1**^**)**					
CIM-616*	9.66 abc	9.70 a	9.62 abcd	9.85 a	9.75 bcd	9.70 cd
GH-Mubarik*	9.68 ab	9.69 ab	9.65 abc	9.70 cd	9.73 bcd	9.67 d
CIM-620**	9.61 bcd	9.65 abc	9.58 cde	9.70 cd	9.76 bc	9.67 d
N-414**	9.55 de	9.67 ab	9.53 e	9.86 a	9.75 bc	9.79 ab
**LSD** (**p ≤ 0.05**)	**0.08**			**0.08**		
	**Available potassium (mg kg**^**-1**^**)**					
CIM-616*	199 abcd	203 a	201 abc	202	203	204
GH-Mubarik*	200 abc	201 abc	196 cde	202	204	201
CIM-620**	197 bcde	202 ab	194 e	202	202	202
N-414**	197 bcde	201 ab	195 de	203	201	200
**LSD** (**p ≤ 0.05**)	**4.87**			**NS**		
	**Available zinc (mg kg**^**-1**^**)**					
CIM-616*	0.77 abc	0.81 a	0.71 d	0.79 abc	0.82 a	0.76 c
GH-Mubarik*	0.78 ab	0.81 a	0.73 cd	0.81 ab	0.82 a	0.77 bc
CIM-620**	0.77 abc	0.79 a	0.73 cd	0.79 abc	0.80 ab	0.76 c
N-414**	0.77 abc	0.81 a	0.74 bcd	0.79 abc	0.81 ab	0.78 bc
**LSD** (**p ≤ 0.05**)	**0.05**			**0.04**		
	**Available iron (mg kg**^**-1**^**)**					
CIM-616*	3.89 b	4.05 a	3.88 bc	3.92 c	4.11 a	3.90 c
GH-Mubarik*	3.82 bcd	4.00 a	3.75 de	3.86 c	4.02 b	3.86 c
CIM-620**	3.79 cde	3.99 a	3.71 e	3.89 c	4.03 b	3.86 c
N-414**	3.82 bcd	4.03 a	3.76 de	3.94 c	4.08 ab	3.89 c
**LSD** (**p ≤ 0.05**)	**0.09**			**0.08**		

* = *Bt* cultivars

** = non-*Bt* cultivars, Means followed by varying letters for an experimental year differ at significantly (p ≤0.05) from each other, NS = Non-significant

Egyptian-clover with *Bt* mulch had the highest EC during both years, whereas the lowest EC was noted for wheat crop with non-*Bt* mulch. The highest soil pH was recorded for wheat crop with *Bt* mulch during both years, while canola crop with non-*Bt* mulch resulted in the lowest soil pH during both the years (Table 5).

The highest available N was recorded for wheat crop with non-*Bt* mulch during both the years. Canola crop with non-*Bt* mulch during both years as well as Egyptian-clover and canola with *Bt* mulch during 2^nd^ study year had the lowest available N. Egyptian-clover with *Bt* mulch during 1^st^ year and wheat crop with both mulch types during 2^nd^ year observed the highest available P. The lowest P was recorded for canola crop with non-*Bt* mulch during 1^st^ year and with both mulch types during 2^nd^ year. The highest available K was recorded for Egyptian-clover with *Bt* mulch, whereas the lowest was noted for canola with non-*Bt* mulch during 1^st^ year. Mulch types and winter crops did not alter the available K during 2^nd^ year (Table 5). The highest available Zn was noted for Egyptian-clover with both mulch types during 1^st^ year and with *Bt* mulch during 2^nd^ year. However, the lowest available Zn was recorded for canola crop with *Bt* and non-*Bt* mulch during 1^st^ and 2^nd^ year, respectively. Like available Zn, the highest available Fe was noted for Egyptian-clover with both mulch types during 1^st^ year and with *Bt* mulch during 2^nd^ year. Canola with non-*Bt* mulch during 1^st^ year, and wheat and canola with both mulch types during 2^nd^ year recorded the lowest available Fe (Table 5).

### Weed dynamics (total weeds’ density m^-2^)

Total weeds density was significantly altered by the interaction among mulch types and winter crops (Table 6). Wheat crop with both mulch types during 1^st^ year had the highest total weed density. Similarly, wheat crop with non-*Bt* mulch had the highest total weed density during 2^nd^ year. Egyptian-clover with *Bt* mulch during both years and canola with non-*Bt* mulch during 1^st^ year had the lowest weed density (Table 6).

**Table 6:** Effect of different mulch types on weed dynamics in different winter crops.

Mulch type	Wheat	Egyptian clover	Canola	Wheat	Egyptian clover	Canola
	2016–17			2017–18		
CIM-616*	97 a	64 ef	74 c	120 ab	82 e	96 d
GH-Mubarik*	90 b	60 g	68 d	107 c	71 f	84 e
CIM-620**	95 a	63 e-g	65 de	124 a	95 d	98 d
N-414**	95 a	62 fg	61 g	115 b	87 e	84 e
**LSD** (**p ≤ 0.05**)	3.29			5.93		

* = *Bt* cultivars

** = non-*Bt* cultivars, Means followed by varying letters for an experimental year differ at significantly (p ≤0.05) from each other

### Morphological and yield parameters of winter crops

#### Wheat

The morphological and yield related attributes of wheat crop were significantly altered by different mulch types during both years except non-significant effect on plant height and number of spikelets per spike (Table 7). The highest values for all morphological and yield-related traits (except for non-significant variables) were noted for the crop with non-*Bt* mulch than *Bt* mulch (Table 7).

**Table 7:** The impact of different mulch types on morphological and yield related traits of wheat crop.

Mulch type	2016–17	2017–18	2016–17	2017–18	2016–17	2017–18	2016–17	2017–18	2016–17	2017–18	2016–17	2017–18	2016–17	2017–18	2016–17	2017–18
	Plant height (cm)		Productive tillers (m^-2^)		Spike length (cm)		Spikelets (spike^-1^)		Grains (spike^-1^)		1000-grain weight (g)		Grain yield (t ha^-1^)		Straw yield (t ha^-1^)	
CIM-616*	95.7	95.4 c	160 b	161 b	12.5 ab	12.8 ab	19.8	20.5	56.1 b	57.3 b	35.9 b	36.4 b	5.90^NS^	6.02 ab	11.4 b	10.2 bc
GH-Mubarik*	96.6	96.8 bc	146 c	149 c	11.8 b	12.2 b	19.9	20.4	55.7 b	56.3 b	34.3 b	36.0 b	5.78	5.94 b	10.9 b	10.0 c
CIM-620**	97.3	97.8 ab	166 ab	164 b	12.2 ab	12.5 ab	20.8	21.3	60.8 a	60.3 a	41.4 a	40.7 a	6.02	6.13 a	11.8 ab	11.4 ab
N-414**	98.2	98.9 a	172 a	173 a	12.8 a	13.1 a	20.9	21.4	59.0 ab	60.3 a	39.0 a	39.7 a	5.96	6.05 ab	12.5 a	11.9 a
**LSD** (**p ≤ 0.05**)	**NS**	**1.8**	**11.17**	**7.56**	**0.78**	**0.78**	**NS**	**NS**	**4.01**	**1.69**	**2.67**	**2.19**	**NS**	**0.16**	**0.90**	**1.21**

* = *Bt* cultivars

** = non-*Bt* cultivars, Means followed by varying letters for an experimental year differ at significantly (p ≤0.05) from each other, NS = Non-significant

### Canola

Different mulch types significantly affected the morphological and yield-related attributes of canola crop during both years except non-significant effect on plant height, plant population and 1000-seed weight (Table 8). The highest values of all morphological and yield-related traits (except for non-significant traits) were noted for the crop sown with non-*Bt* mulch than *Bt* mulch (Table 8).

**Table 8:** The effect of different mulch types on morphological and yield related parameters of canola crop.

Mulch type	2016–17	2017–18	2016–17	2017–18	2016–17	2017–18	2016–17	2017–18	2016–17	2017–18	2016–17	2017–18
	Plant height (cm)		Plant population (m^-2^)		Silique (plant^-1^)		Seeds (silique^-1^)		1000-seed weight (g)		Seed yield (kg ha^-1^)	
CIM-616*	139	139	21.0	21.7	97.3 b	98 b	26.3 b	27.0 b	2.87	2.85	1620 c	1720
GH-Mubarik*	142	141	20.3	21.0	107 ab	108 a	27.2 ab	27.2 b	2.97	2.90	1850 b	1880
CIM-620**	143	142	21.7	22.7	106 ab	109 a	28.1 ab	28.5 ab	2.98	2.94	1970 ab	1920
N-414**	142	141	22.0	23.0	111 a	114 a	29.0 a	29.7 a	2.99	2.94	2070 a	1930
**LSD** (**p ≤ 0.05**)	**NS**	**NS**	**NS**	**NS**	**9.94**	**8.04**	**1.80**	**2.40**	**NS**	**NS**	**128.96**	**NS**

* = *Bt* cultivars

** = non-*Bt* cultivars, Means followed by varying letters for an experimental year differ at significantly (p ≤0.05) from each other, NS = Non-significant

### Egyptian-clover

Different mulch types significantly affected the morphological and yield related attributes of Egyptian-clover during both years except non-significant effect on plant height (Table 9). The highest values of all morphological and yield-related traits (except for non-significant traits) were noted for the crop sown with non-*Bt* mulch than *Bt* mulch (Table 9).

**Table 9:** Effect of different mulch types on morphological and yield related traits of Egyptian clover.

Mulch type	2016–17	2017–18	2016–17	2017–18	2016–17	2017–18	2016–17	2017–18
	Plant population (m^-2^)		Final Plant height (cm)		Total fodder weight (t ha^-1^)		Crude protein content (%)	
CIM-616*	60.0	58.9	62.8 c	61.8 c	29.2 b	30.1 c	21.2 b	20.0 b
GH-Mubarik*	53.3	56.8	64.8 b	62.6 c	27.6 b	30.8 bc	21.2 b	20.9 b
CIM-620**	66.0	69.4	66.4 ab	69.2 a	34.7 a	33.1 a	24.0 a	23.6 a
N-414**	61.7	65.1	67.2 a	67.5 b	32.3 a	31.9 ab	24.4 a	24.5 a
**LSD** (**p ≤ 0.05**)	**NS**	**NS**	**1.82**	**1.00**	**2.67**	**1.52**	**1.38**	**1.58**

* = *Bt* cultivars

** = non-*Bt* cultivars, Means followed by varying letters for an experimental year differ at significantly (p ≤0.05) from each other, NS = Non-significant

## Discussion

### Soil properties

Wheat crop observed the highest soil porosity and penetration resistance. Mulching of *Bt*-cotton increased soil EC compared to non-*Bt* mulches. The highest EC and pH were noted in the plots of Egyptian-clover and wheat with any mulch type. The inclusion of leguminous crops in cropping system improve soil physical properties by lowering soil compaction [49–52]. However, the results of this study are contrasting as no improvement was noted with Egyptian-clover. It has been reported that mulching can reduce water evaporation and salt accumulation in soil, which eventually reduce soil EC [53]. Mulching non-*Bt* cotton lead to the reduction in the accumulation of soluble salts in the soil surface, which lowered the EC of the soil. On the other hand, addition of *Bt* toxin released from *Bt* mulches enhanced soil EC. The thickness of applied mulches significantly alters soil pH [54, 55], by adding or conserving organic matter and acids coming from the rotten plant debris [56].

Higher availability of soil nutrients like N, P and Fe was observed with *Bt* mulch (Table 5). Wheat and Egyptian-clover had the highest available N, P, K, Zn and Fe (Table 5). Introduction of *Bt*-crops or their mulches in the fields can alter nutrient cycling. This may be due to products of introduced genes or by modification rhizosphere chemistry [57]. Different studies have confirmed that any variation in root exudates, particularly during addition of new genetic trait affects several processes, including mineral nutrition [58, 59]. This reveals that *Bt* toxin can alter root exudates and microbe’s colony, which have significant influence on nutrients dynamics in soil. Moreover, *Bt*-cotton reduces the available N and K, while increases Zn and P [25, 26].

### Weed dynamics

Mulching non-*Bt* cotton resulted in higher weed infestation than *Bt* mulches (Table 6). Similarly, wheat crop observed the highest weed infestation compared to the rest of winter crops. Weed infestation plays key role in crop productivity. Mulching has been found a viable option for weed control as straw mulching reduces weed emergence and growth [60–64]. Transgenic *Bt*-cotton produces *Bt*-toxins (*Cry* proteins) which may accumulate and persist in soil due to their binding ability on soil components. Although there are no known mechanisms, *Bt* toxins significantly affect weed dynamics [18, 20]. The non-*Bt* mulches observed higher weed infestation because of the absence of *Bt* toxins. Nonetheless, low availability of nutrients in non-*Bt* mulched plots indicated that both winter crops and weeds consumed these nutrients.

Allelopathic nature of crops such as wheat [65] and canola [66, 67] could lower weed density. However, higher weed density was observed in these crops than Egyptian-clover, which is not considered as an allelopathic crop. Egyptian-clover was sown through broadcast method, which gave weeds less space for infestation [3]. The wheat crop observed higher weed density due to the availability of more space for weed infestation compared to Egyptian-clover.

### Morphological and yield related attributes

Non-*Bt* mulches caused more improvement in morphological and yield-related traits of all winter crops compared to *Bt* mulches. The *Bt* crops release *Bt* toxins, which alter enzymatic activities and nutrient availability. Thus, reduced nutrient availability along with toxins’ effect probably resulted in weak morphological and yield-related traits of crops grown with *Bt* mulches.

The improved performance of winter crops with non-*Bt* mulches can be attributed to low concentration of *Bt* toxin in the soil. Various studies proved that mulching conserves water and control weeds, which increase crop productivity [68–70]. The non-*Bt* mulches resulted in better soil conditioning (maximum soil porosity and organic matter content) than *Bt* mulches. Organic matter is a rich source of nutrients to crop plants. This may increase absorption efficiency, resulting in elevated crop productivity [71]. Continuous sowing of *Bt*-cotton on a similar field can increase *Bt* toxins in the soil, which can alter the activity and composition of the soil microbes [27, 72–75]. It has also been shown that non-*Bt* crop extracts improved biochemical nature of leaf by increasing chlorophyll b, dissolvable sugars and catalase development in subsequent wheat crop [76]. This shows that non-*Bt* mulches improve water conservation, soil physical properties, add organic matter and result in higher productivity.

## Conclusion

The *Bt* and non-*Bt* mulches differentially affected soil properties, weed dynamics and productivity of winter crops. Overall, non-*Bt* mulches had better impact on the measured traits than *Bt* mulches. The toxins released by *Bt* mulches lowered weed density; however, negatively influenced soil properties and productivity of winter crops. Therefore, appropriate crop rotation measures should be opted for the soils under *Bt*-cotton cultivation for soil conservation and yield sustainability of crops following cotton. Nonetheless, non-*Bt* mulches can be used for improving soil properties and performance of winter crops.
